The article "Study on PD-L1 Expression in NSCLC Patients and Related Influencing Factors in the Real World" was retracted in 2023. Reasons: suspected computer-generated content; unreliable results or conclusions; concerns about the data; concerns about the results or conclusions.

# Study on PD-L1 Expression in NSCLC Patients and Related Influencing Factors in the Real World

**DOI:** 10.1155/2021/3273347

**Published:** 2021-12-28

**Authors:** Yefei Zhu, Shuangxiang Lin, Yueping Wang, Bingxiao Shen, Ling Lin, Liangxing Wang, Susu He

**Affiliations:** ^1^Department of Respiratory Medicine, Tai Zhou Hospital of Zhejiang Province Affiliated to Wenzhou Medical University, Linhai, Zhejiang, China; ^2^Department of Radiology, Tai Zhou Hospital of Zhejiang Province Affiliated to Wenzhou Medical University, Linhai, Zhejiang, China; ^3^Department of Geriatrics, Tai Zhou Hospital of Zhejiang Province Affiliated to Wenzhou Medical University, Linhai, Zhejiang, China; ^4^Department of Respiratory Medicine, The First Affiliated Hospital of Wenzhou Medical University, Wenzhou, Zhejiang, China

## Abstract

PD-L1 is one of the current biomarkers for immune checkpoint inhibitor (ICI) therapy in patients with non-small-cell lung cancer. However, the expression of PD-L1 in the real world and its related influencing factors remain unclear. We want to observe the expression of PD-L1 in the real world and study the related influencing factors through the collection and analysis of clinical data. R software (version 4.0) was used to perform data analysis and the “corplot” package for correlation analysis. A total of 296 individuals (mean [SD] age, 67 [9] years; 23%female) were assessed. According to the expression amount of PD-L1, the cohort was divided into low nonexpression group (PD‐L1 < 1%, 26.7%), low-expression group (1% ≤ PD‐L1 < 50%, 49.3%), and high-expression group (PD‐L1 ≥ 50%, 23.5%). Age, gender, underlying diseases, smoking status, and PD-L1 expression level were not statistically significant. We found that the expression of PD-L1 was correlated with serum albumin (*P* < 0.05) and pathological type (*P* < 0.05) and had a negative correlation with EGFR mutation but did not correlate with gender, age, smoking status, combined with underlying diseases, tumor stage, whether it was initially treated or not, sampling site, specimen type, specimen storage time, R-IFN, CD4, CD8, NLR, CRP, and LDH. The present findings indicated that serum albumin, pathological type, and EGFR mutations are associated with PD-L1 expression in patients with NSCLC, which may provide a new basis for individualized immunotherapy and need further study to confirm. The results of this study help to further reveal the actual expression of PD-L1 in non-small-cell lung cancer patients with real events.

## 1. Introduction

Lung cancer is one of the leading causes of cancer morbidity and death worldwide. According to the latest statistics, lung cancer occupies second place (about 11.4%) of new cancers worldwide in 2020 and is the main cause of cancer death [1]. Among lung cancer patients, non-small-cell lung cancer (NSCLC) accounts for about 85% [2].

The article "Study on PD-L1 Expression in NSCLC Patients and Related Influencing Factors in the Real World" was retracted in 2023. Reasons: suspected computer-generated content; unreliable results or conclusions; concerns about the data; concerns about the results or conclusions.

In recent years, different treatment options have emerged for specific cell types of NSCLC. Targeted therapies with targeted driver gene mutations are used as first-line therapy for advanced NSCLC [3]. Patients can benefit greatly from targeted therapies. However, these patients only account for a small proportion of NSCLC patients [3, 4]. For a long time in the past, the majority of patients who were not found to be positive for driver genes relied mainly on traditional chemotherapy to improve prognosis. In recent years, immunotherapy has become increasingly popular due to its outstanding efficacy [5]. The Food and Drug Administration (FDA) has approved the use of a variety of immune checkpoint inhibitors (ICIs), mainly based on the improvement of patients' OS compared with chemotherapy [6–10]. Although the emergence of immune checkpoint inhibitors has changed the traditional cancer treatment strategy and brought more opportunities to cancer patients, in patients with advanced NSCLC, the overall response rate is poor [6–10], which may be mainly due to the lack of a precise biomarker to screen patients suitable for immune checkpoint inhibitor therapy.

As one of the biomarkers of immune checkpoint inhibitor (ICI) therapy, programmed cell death-ligand 1 (PD-L1) has entered the clinical practice of non-small-cell lung cancer. At present, a large number of clinical trials have proved that patients with high expression of PD-L1 often have better efficacy of immune checkpoint inhibitors [6–10], but PD-L1-negative patients can also benefit [1]. One of the reasons for this may be that these clinical trials have certain standards and requirements for tissue collection and selection, which cannot fully reflect the actual situation of PD-L1 expression in the real world. In the “real world,” tumor samples have greater variability and more heterogeneity of clinical, pathological, and molecular characteristics [10, 11]. Holmes et al. [11] showed that the expression of PD-L1 was different in patients with different driver gene mutations. Currently, few studies have evaluated whether clinical features affect PD-L1 expression and whether tumor sampling procedures, such as sample type (e.g., biopsy and resection), sample site, and prior antitumor therapy affect PD-L1 expression [12, 13]. The purpose of this study was to observe the expression of PD-L1 in NSCLC in the real world and to investigate its influencing factors, including clinical features, tumor type, histological subtypes, driver gene mutations, and prior antitumor therapy.

The article "Study on PD-L1 Expression in NSCLC Patients and Related Influencing Factors in the Real World" was retracted in 2023. Reasons: suspected computer-generated content; unreliable results or conclusions; concerns about the data; concerns about the results or conclusions.

## 2. Materials and Methods

### 2.1. Patient Information

We collected 296 patients with NSCLC who underwent PD-L1 testing at Taizhou Hospital in Zhejiang Province between April 1, 2018, and June 1, 2021, and their clinical characteristics. Clinical features including the detection of age, sex, smoking history, with basic diseases, cancer stage (International Association for the Study of Lung Cancer version 8 lung cancer TNM staging) [14], histology, driving cancer gene mutation status, serum neutrophil count/lymphocyte count (neutrophil and lymphocyte ratio, NLR), serum albumin, and serum albumin (propagated) are obtained from the electronic patient records. This study protocol is in line with the Helsinki Declaration and approved by the Ethics Committee of Taizhou Hospital in Zhejiang Province. Informed consent is not required based on the retrospective analysis of anonymous patient data.

### 2.2. PD-L1 Immunohistochemical Detection

The main instruments were Dako Autostainer Link 48 automatic immunohistochemical staining instrument and the automatic immunohistochemical pretreatment instrument (PT Link, PT200). According to the manufacturer's recommended method, PDA-L1 was stained with pharmDx antibody (Clone 22C3, Dako North America, Inc., Agilent/Dako, Carpinteria, CA, USA) for immunohistochemical staining.

### 2.3. Mutation Tests

Tumor tissue samples from all patients were fixed with 10% neutral formalin buffer and paraffin embedded. Driver gene variation detection: DNA and RNA extraction was done using FFPE DNA/RNA kit (Ed Bio). Mutations in 9 driver genes including EGFR, ALK, ROS1, RET, KRAS, BRAF, PIK3CA, HER2, and MET were detected by a multigene detection kit (fluorescence PCR) (Eddard).

### 2.4. Interpretation of Results

All sections were reviewed by two experienced pathologists for PD-L1 results. If the independent opinions are not consistent, the two doctors should review and discuss together to reach a unanimous judgment. According to the tumor proportion score (TPS) of PD-L1 expression in tumor cells to tumor nests, the tumor cells were divided into three groups: no expression (PD‐L1 < 1%), low expression (1% ≤ PD‐L1 < 50%), and high expression (PD‐L1 ≥ 50%).

### 2.5. Statistical Analysis

Descriptive statistics are reported as means ± standard or medians with interquartile ranges for continuous variables and frequencies with percentage for classified variables. R software (version 4.0) was used to state analysis, and the “corplot” package was used for correlation analysis. *χ*^2^ test, *T*-test, or Mann–Whitney *U* test was used to compare the continuous variables, and skewness and kurtosis were used to test the normality. *P* < 0.05 was statistically significant.

The article "Study on PD-L1 Expression in NSCLC Patients and Related Influencing Factors in the Real World" was retracted in 2023. Reasons: suspected computer-generated content; unreliable results or conclusions; concerns about the data; concerns about the results or conclusions.

## 3. Results

### 3.1. Basic Features

A total of 296 patients with NSCLC were enrolled in the study. There were 226 males (76.3%) and 69 females (23.7%) with an average age of 67.21 ± 9.3 years. According to tumor PD-L1 expression stratification, there were 79 patients (26.7%) in the nonexpression group, 146 patients (49.3%) in the low-expression group, and 70 patients (23.5%) in the high-expression group. Age, gender, underlying diseases, smoking status, and PD-L1 expression level were not statistically significant. The specific clinical characteristics of the patients are shown in Table 1.

### 3.2. Clinical Test Data

For the patient's clinical inspection, data including interferon-gamma (r-IFN), CD4, CD8, NLR, C-reactive protein (CRP), and propagated for data statistics show that patients with serum albumin level and the expression of PD-L1 exist difference (*P* < 0.05); serum albumin level was significantly higher in the high-expression group and the low-expression group does not express, and there is the difference (*P* < 0.05). There were no significant differences in r-IFN, CD4, CD8, NLR, CRP, and LDH among different expression groups. See Table 2.

### 3.3. Tumor Sampling Characteristics

256 patients (86.5%) were initially treated and 38 patients (12.8%) were treated, and there was no statistical significance in the PD-L1 group. 244 patients (83.5%) were sampled from primary lesions and 52 patients (16.5%) from metastatic lesions, including 32 cases of lymph nodes (10.8%), 13 cases of pleural fluid (13%), and 7 cases of other metastatic lesions (2.36%). CT-guided lung puncture and tracheoscopic biopsy were the main methods of sampling, showing no statistical difference with PD-L1 expression. In the storage time analysis of PD-L1 samples, the average storage time of the nonexpression group was 51 days, that of the low-expression group was 67.6 days, and that of the high-expression group was 45.1 days, showing no statistical significance. See Table 3.

### 3.4. Tissue Types and Driver Gene Mutations

There were 149 cases of squamous cell carcinoma, 131 cases of adenocarcinoma, and 15 cases of other non-small-cell lung cancer, accounting for 34%, 59%, and 6% of the nonexpression group, 58%, 39%, and 3% of the low-expression group, and 54%, 39%, and 7% of the high-expression group, respectively. The expression of PD-L1 in different pathological types had statistical significance (*P* < 0.05). In adenocarcinoma, the expression rate of the low-expression group was higher than that of the nonexpression group and the high-expression group, with statistical significance (*P* < 0.05), as shown in Table 4.

The article "Study on PD-L1 Expression in NSCLC Patients and Related Influencing Factors in the Real World" was retracted in 2023. Reasons: suspected computer-generated content; unreliable results or conclusions; concerns about the data; concerns about the results or conclusions.

Among 111 patients with oncogene mutation, 30.4% had epidermal growth factor receptor (EGFR) mutation and 12.6% had other gene mutations. In the low-expression group, EGFR mutation accounted for 15.6%, ALK mutation accounted for 2.04%, and other gene mutation accounted for 12.6%. In the high-expression group, EGFR mutations accounted for 20%, and other gene mutations accounted for 17.1%, as shown in Figure 1.

Correlation analysis of patients with EGFR gene mutation showed that there was a negative correlation between the nonexpression group, the low-expression group, and the high-expression group, and the correlation coefficients were -0.6, -0.14, and -0.55, respectively, suggesting that EGFR mutation was negatively correlated with PD-L1 expression. No clear association was found for the remaining mutations, as shown in Figure 1.

### 3.5. Choice of the Treatment Plan

For analysis of treatment options for patients with advanced driver gene negative non-small-cell lung cancer, immunotherapy began to rise gradually in our hospital in 2019, and with the increase of time, the number of patients selected for immunotherapy regimen gradually increased, and the proportion of patients in the high-expression group gradually increased, as shown in Figure 2.

## 4. Discussion

At present, PD-L1 is one of the biomarkers for non-small-cell lung cancer patients to choose immune checkpoint inhibitor (ICI) therapy, in which the expression of PD-L1 is used as a prognostic indicator for NSCLC patients receiving palivizumab therapy [15], but the expression of PD-L1 and its related influencing factors in the real world is still unclear. In the “real world,” tumor samples have greater variability and more heterogeneity of clinical, pathological, and molecular characteristics [10, 11]. The purpose of this study was to observe the expression of PD-L1 in the real world and evaluate whether clinical features affected the expression of PD-L1. Make the clinical application of PD-L1 detection and its role in guiding treatment decisions more meaningful.

At present, in different clinical trials, PD-L1 antibodies of different manufacturers are used by different pharmaceutical manufacturers and tested on different platforms [6–10], as shown in Table 5. Therefore, the expression results of PD-L1 obtained lack comparability. Tsao et al. [16] showed similar expressions of Dako 28-8, Dako 22C3, and Ventana SP263 in the detection of non-small-cell lung cancer. However, the results of Ventana SP142 were inconsistent, which may underestimate the high positive rate of PD-L1. Wang et al. [12] also confirmed the difference in PD-L1 expression measured by antibodies from different sources, and the study also showed that different operators would affect the detection results. Lloyd et al. [17] showed that the immunocytochemical staining results of PD-L1 were affected by different solution reagents, so strict validation of different forms of cell smear in PD-L1 detection was required, including collection and fixation of specimen materials and interpretation of results. To ensure the feasibility of the test and the accuracy of the results, the “PD-L1” (22C3) detection kit (immunohistochemical method) of Dako North America and the Dako Autostainer Link 48 immunohistochemical staining instrument was used in this study, and the interpretation of the results was carried out in strict accordance with the standards [18]. To avoid the difference of interpretation results among different physicians and influence the choice of the treatment plan, this study was conducted by two fixed experienced pathologists who interpreted together. Among the 296 NSCLC patients, the nonexpression group, the low-expression group, and the high-expression group accounted for 26.7%, 49.3%, and 23.5%, respectively, which is similar to the study of Ye et al., the non-expression group accounted for 27%, the low-expression group 40.3%, and the high-expression group 27.5% [19]. In the process of actual clinical diagnosis and treatment, on the one hand, we hope to get the correlation between different detection antibody consistency [20] and research results; on the other hand, we also hope to strengthen the standardized testing in clinical practice, the strict uniform interpretation standards, and the pathologist interpretation standards of training; it will make the clinical application of PD-L1 testing more meaningful in guiding treatment decisions.

The article "Study on PD-L1 Expression in NSCLC Patients and Related Influencing Factors in the Real World" was retracted in 2023. Reasons: suspected computer-generated content; unreliable results or conclusions; concerns about the data; concerns about the results or conclusions.

At present, some studies have shown that smoking can increase the expression of PD-L1 in NSCLC patients [21]. This may be due to tobacco carcinogens that cause mutations in tumor occurrence, causing a more new antigen and the increase of the PD-L1 expression, and in addition, smoking can induce inflammation, including T cells and inflammatory cytokines, such as interferon-g, and can raise PD-L1 expression [21], but this research shows smoking status in patients with no statistical difference with PD-L1 expression, requiring a larger sample size study to confirm further.

Serum albumin is often used as an indicator of a patient's nutritional status. Studies have shown that serum albumin level can be an important predictor and prognostic indicator for NSCLC patients treated with immune checkpoint inhibitors, especially in patients with PD-L1 TPS ≥ 50% [22]. Studies have shown that nutritional status plays an important determinant in the process of the immune response, and malnutrition often leads to immune deficiency in patients, which leads to impaired cell-mediated antitumor immune function [23]. Thus, a patient's nutritional status may influence the tumor microenvironment and thus the response to immune checkpoint inhibitors. This research detecting PD-L1 albumin index during the same period found that a difference exists in serum albumin level and the expression of PD-L1 (*P* < 0.05), serum albumin level was significantly higher in the high-expression group but not expressed in the low-expression group, and there is the difference (*P* < 0.05), but whether it can prompt the curative effect of immunotherapy needs further study.

Previous studies have shown that the difference in PD-L1 expression between primary tumor and local lymph node metastasis is relatively small [24, 25]. However, some studies have found that middle and advanced tumors are more likely to express PD-L1 than early tumors [13, 26], and the expression of PD-L1 in lymph node tissues is higher than that in other metastatic sites such as brain and bone [13]. Uruga et al. and Zhou et al. have also confirmed that the expression of PD-L1 in distant metastatic NSCLC is different from that in primary NSCLC, suggesting intratumor heterogeneity of PD-L1 expression [27, 28]. At present, it is not clear why there is a difference in the expression of PD-L1 between the metastatic sites, and further research is needed. However, in this study, there was no statistical significance between whether the samples were collected from the primary foci and the expression of PD-L1, which may be due to the small sample size of the metastatic foci. In clinical practice, specimens of primary foci and metastatic foci are often not obtained at the same time. According to previous studies, clinicians should try to avoid other prediction sites with less reliable PD-L1 expression, such as bone, when obtaining specimens.

Most immunotherapy clinical trials currently use histological specimens for quantitative detection of PD-L1. Studies have shown that the expression level of PD-L1 in histological specimens is significantly different from that of the whole surgically resected tumor tissue specimens [29], which may be related to the number of biopsies and tumor area [30]. Therefore, to meet the actual clinical requirements, sufficient tissue specimens should be obtained to reduce the difference in detection results [31]. However, in the real world, cytological specimens are selected for patients with advanced NSCLC and for patients with difficulty in obtaining histological specimens. In this study, most of the specimens were histological specimens (92.2%) and a small part was cytological specimens (4.39%). The samples obtained only accounted for a small part of the entire tumor tissue, and the specimen types showed no statistical significance for the expression of PD-L1. However, Pak et al. and Lozano et al. and other studies confirmed the feasibility and effectiveness of cytological specimens for quantitative detection of PD-l1, and the consistency rate with surgical specimens reached 81.1%~97.3% [32, 33]. Therefore, cytological specimens can be selected when it is difficult to obtain tissue samples, but large-scale studies and standardized procedures for cell collection are required before they can be included in routine clinical use.

The article "Study on PD-L1 Expression in NSCLC Patients and Related Influencing Factors in the Real World" was retracted in 2023. Reasons: suspected computer-generated content; unreliable results or conclusions; concerns about the data; concerns about the results or conclusions.

Previous studies have shown that paraffin blocks fixed with formalin can preserve proteins for decades, and sample age is unlikely to affect PD-L1 expression by reducing antigenic stability [34]. This is similar to our study. However, some studies have shown that the storage time of specimens will affect the expression of PD-L1, and archived specimens over 3 years will affect the detection results of PD-L1 [35]. Several studies have shown that PD-L1 glycosylation exists on the surface of various types of cancer cells (including lung cancer, melanoma, and breast cancer), which affects the structure and function of proteins and causes their polypeptide antigens to be unable to be recognized by PD-L1 antibodies, affecting the immunohistochemical detection of specimens and leading to abnormal results [36]. Boothman et al. [21] also found that fresh biopsy specimens can more accurately assess current tumor PD-L1 expression, and archived samples may show low/negative expression results. Whether this difference has a certain clinical significance remains to be confirmed by further studies. Studies have shown that when low/negative expression results occur in archived samples, new biopsy specimens can be retrieved to more accurately assess the current state of tumor PD-L1 expression, especially if the patient has previously received chemotherapy or radiotherapy [21].

The study of Boothman et al. [21] showed that the expression of PD-L1 in squamous carcinoma was higher than that in nonsquamous carcinoma. In the CHECKMATE 057 clinical trial of patients with nonsquamous cell carcinoma, both the PD-L1-positive group and the PD-L1-negative group showed benefit from second-line treatment with natalizumab, while the CHECKMATE 017 clinical trial suggested that the expression of PD-L1 could not predict the PFS and OS of natalizumab, which may be caused by the different histological types of the two patients [4]. Our study also found different pathological types of PD-L1 expression differences, among which 149 were squamous carcinoma, 131 cases of adenocarcinoma, and other non-small-cell lung cancer, 15 cases among them, respectively, squamous carcinoma in the nonexpression group was 34%, 59%, and 6%, in the low-expression group 58%, 39%, and 3%, and in the high-expression group 54%, 39%, and 7% (*P* < 0.05); adenocarcinoma expression rate in the low-expression group is higher than that in the nonexpression group and the high expression group, with statistical significance (*P* < 0.05). Current data show that tumor driver gene mutations are closely associated with abnormal activation of PD-1/PD-L1 signaling. A global, multicentre, retrospective observational (EXPRESS) study found a relationship between PD-L1 expression and molecular biomarkers, including EGFR mutations and ALK translocations [37]. In this study, correlation analysis of EGFR gene mutation showed that EGFR mutation was negatively correlated with PD-L1 expression, but due to the small number of patients with ALK mutation, the correlation could not be further analyzed. Lee et al. also found a negative correlation between PD-L1 expression and EGFR mutations in cohort analysis of Asian non-small-cell lung cancer patients [38]. But the current mechanism is unclear. This finding implies that patients with different tissue types and driver gene mutations may benefit differently from ICI treatment, which needs to be demonstrated in further studies.

The article "Study on PD-L1 Expression in NSCLC Patients and Related Influencing Factors in the Real World" was retracted in 2023. Reasons: suspected computer-generated content; unreliable results or conclusions; concerns about the data; concerns about the results or conclusions.

Studies have shown that the expression of PD-L1 in the neoadjuvant chemotherapy group is higher than that in the nonneoadjuvant chemotherapy group, which may be due to the activation of the specific immune response mechanism of lung cancer, resulting in the upregulation of PD-L1 expression [21, 39]. At the same time, studies have also shown complex changes in PD-L1 expression after treatment with tyrosine kinase inhibitor (TKI), in which 21.3% of cases were increased and 19.1% were decreased [40]. The expression of PD-L1 was significantly decreased after immunotherapy compared with untreated or other antitumor therapies [36]. These studies have shown that PD-L1 changes are associated with different tumor treatments. However, in this study, no correlation was found between primary treatment and retreatment and PD-L1 expression, so further clinical data is needed to confirm and provide guidance for the dynamic monitoring of PD-L1 expression as a treatment option.

In our study, we found that for patients with negative late-stage driver genes, the selection of immunotherapy options increased year by year. Previously, patients with lung cancer preferred chemotherapy alone, which may be due to economic constraints. The introduction of innovative high-cost drugs in clinical treatment, such as the application of ICIs in the treatment of lung cancer, has caused certain social concerns and economic problems. Accordingly, in the United States, in 2020, the cost of cancer treatment is expected to be up to 173 billion dollars [41]; along with the growing economic burden of cancer treatment, the clinical thinking of clinical benefit and toxicity of treatment costs at the same time also gradually becomes one of the factors, because the cost-benefit analysis is to assess whether new interventions at a reasonable cost to provide clinical benefit is an important strategy, which has a significant influence on health policy and public policy [42]. Verma et al. proposed that pembrolizumab was cost-effective in NSCLC, while nivolumab was not through systematic analysis [43]. In a systematic review and meta-analysis, Ding et al. found that pembrolizumab first-line treatment in more than 50% of patients was more cost-effective than platinum-based chemotherapy and proposed that drug discounts or the use of PD-L1 expression as biomarkers could improve the cost-effectiveness of immunotherapy [44]. In 2021, some companies in China will readjust the price of ICIs according to the actual situation and some ICIs will be included in the medical insurance. In the real world, more patients will choose immune-related drug treatment. It will be further confirmed that the selection of drugs related to immune checkpoint inhibitors based on the expression of PD-L1 will improve the cost-effectiveness.

The article "Study on PD-L1 Expression in NSCLC Patients and Related Influencing Factors in the Real World" was retracted in 2023. Reasons: suspected computer-generated content; unreliable results or conclusions; concerns about the data; concerns about the results or conclusions.

This study is a retrospective study with a small sample size of rare driver gene mutations, and the clinical efficacy of antitumor therapy has not been tracked yet, which requires multicenter and further follow-up study.

## 5. Conclusion

In conclusion, this real-world study found that serum albumin, pathological type, and EGFR mutations were associated with PD-L1 expression in patients with NSCLC, which may provide a new basis for individualized immunotherapy. The sample size of some rare gene mutations is small, which needs to be confirmed by further large sample data. This study helps to further reveal the actual expression of PD-L1 in non-small-cell lung cancer patients with real events.

## Figures and Tables

**Figure 1:** Correlation between driver gene mutation and PD-L1 expression in patients with non-small-cell lung cancer.

**Figure 2:** Treatment options for patients with advanced driver gene negative non-small-cell lung cancer.

**Table 1:** Correlation between patient clinical features and tumor PD-L1 expression.

	PD‐L1 < 1% (*n* = 79)	1% ≤ PD‐L1 < 50% (*n* = 147)	PD‐L1 ≥ 50% (*n* = 70)	*P* value	OR
Age	67.18 ± 9.3	67.01 ± 9.03	67.46 ± 9.54	0.863	0.147
Sex				0.218	3.051
Male	58 (73%)	119 (81%)	50 (71%)		
Female	21 (27%)	28 (19%)	20 (29%)		
Diseases of the blood system				0.734	Fisher
Absent	79 (100%)	144 (99%)	70 (100%)		
Present	0 (0%)	2 (1%)	0 (0%)		
Diabetes				0.109	4.431
Absent	68 (86%)	137 (94%)	61 (87%)		
Present	11 (14%)	9 (6%)	9 (13%)		
Diseases of the central system				0.912	Fisher
Absent	73 (92%)	136 (93%)	66 (94%)		
Present	6 (8%)	10 (7%)	4 (6%)		
Rheumatic immune disease				0.518	Fisher
Absent	78 (99%)	142 (97%)	70 (100%)		
Present	1 (1%)	4 (3%)	0 (0%)		
Heart disease				0.415	1.761
Absent	45 (57%)	96 (66%)	45 (64%)		
Present	34 (43%)	50 (34%)	25 (36%)		
Other cancer				0.771	Fisher
Absent	75 (95%)	138 (95%)	68 (97%)		
Present	4 (5%)	8 (5%)	2 (3%)		
COPD				0.743	0.594
Absent	68 (86%)	122 (84%)	57 (81%)		
Present	11 (14%)	24 (16%)	13 (19%)		
Other diseases				0.966	0.07
Absent	72 (91%)	132 (90%)	64 (91%)		
Present	7 (9%)	14 (10%)	6 (9%)		
Chronic kidney disease				0.317	Fisher
Absent	77 (97%)	145 (99%)	70 (100%)		
Present	2 (3%)	1 (1%)	0 (0%)		
Smoking status				0.245	2.812
No	37 (47%)	54 (37%)	32 (46%)		
Yes	42 (53%)	93 (63%)	38 (54%)		

COPD: chronic obstructive pulmonary disease.

The article "Study on PD-L1 Expression in NSCLC Patients and Related Influencing Factors in the Real World" was retracted in 2023. Reasons: suspected computer-generated content; unreliable results or conclusions; concerns about the data; concerns about the results or conclusions.

**Table 2:** Correlation between patient clinical test data and tumor PD-L1 expression.

	PD‐L1 < 1% (*n* = 79)	1% ≤ PD‐L1 < 50% (*n* = 147)	PD‐L1 ≥ 50% (*n* = 70)	*P* value
R-interferons (pg/mL)	1.75 (0.95)	1.79 (1.48)	1.32 (0.53)	0.634
CD4 (%)	33.64 (10.59)	38.57 (8.73)	32.81 (16.03)	0.447
CD8 (%)	20.82 (8.99)	25.68 (11.40)	17.19 (7.37)	0.137
NLR (%)	4.08 (4.11)	4.42 (3.12)	4.34 (3.18)	0.771
CRP (mg/L)	27.62 (39.29)	26.67 (41.28)	38.05 (43.80)	0.188
Propagated (g/L)	39.51 (5.41)	37.37 (5.36)	37.52 (4.92)	0.014
LDH (U/L)	242.82 (218.95)	201.13 (107.23)	226.38 (166.00)	0.254

NLR: ratio of neutrophil count to lymphocyte count; CRP: C-reactive protein; LDH: lactate dehydrogenase.

**Table 3:** Correlation between tumor sampling characteristics of patients and PD-L1 expression.

	PD‐L1 < 1%	1% ≤ PD‐L1 < 50%	PD‐L1 ≥ 50%	ALL	*P* value
	(*n* = 79)	(*n* = 147)	(*n* = 70)	*N* = 296	
Sampling method					0.485
Ultrasound puncture	1 (1.27%)	11 (7.48%)	5 (7.14%)	17 (5.74%).	
CT puncture	34 (43.0%)	45 (30.6%)	25 (35.7%)	104 (35.1%)	
Ultrasonic tracheoscope	8 (10.1%)	12 (8.16%)	3 (4.29%)	23 (7.77%)	
Bronchoscope	29 (36.7%)	69 (46.9%)	29 (41.4%)	127 (42.9%)	
Operation	3 (3.80%)	4 (2.72%)	3 (4.29%)	10 (3.38%)	
Chest puncture	3 (3.80%)	5 (3.40%)	5 (7.14%)	13 (4.39%)	
Thoracoscope	1 (1.27%)	1 (0.68%)	0 (0.00%)	2 (0.68%)	
Specimen type					0.676
Organization	73 (92.4%)	138 (93.9%)	62 (88.6%)	273 (92.2%)	
Cells	3 (3.80%)	5 (3.40%)	5 (7.14%)	13 (4.39%).	
Surgical specimens	3 (3.80%)	4 (2.72%)	3 (4.29%)	10 (3.38%)	
Sampling position					0.923
Primary tumor	66 (83.5%)	121 (82.3%)	57 (81.4%)	244 (82.4%)	
Lymph node	8 (10.1%)	17 (11.6%)	7 (10.0%)	32 (10.8%)	
Pleural effusion	3 (3.80%)	5 (3.40%)	5 (7.14%)	13 (4.39%)	
Other metastases^1^	2 (2.53%)	4 (2.72%)	1 (1.43%)	7 (2.36%)	
Treatment or not^2^					0.986
Treatment-naive^3^	69 (87.3%)	126 (85.7%)	61 (87.1%)	256 (86.5%)	
Retreatment^4^	9 (11.4%)	20 (13.6%)	9 (12.9%)	38 (12.8%)	
Unknown^5^	1 (1.27%)	1 (0.68%)	0 (0.00%)	2 (0.68%)	
TNM					0.486
I	4 (5.06%)	4 (2.72%)	1 (1.43%)	9 (3.04%)	
II	2 (2.53%)	4 (2.72%)	1 (1.43%)	7 (2.36%)	
III	21 (26.6%)	56 (38.1%)	21 (30.0%)	98 (33.1%)	
IV	52 (65.8%)	83 (56.5%)	47 (67.1%)	182 (61.5%)	
Specimen storage time^6^	51.0 (133)	67.6 (187)	45.1 (113)	44.5 (93.4)	0.43

TNM: stage of lung cancer, International Association for the Study of Lung Cancer 8th edition. ^1^Other metastases: except lymph nodes, pleural effusion, and other metastases, such as bone. ^2^Whether the patient received antitumor therapy at the time of PD-L1 test. ^3^The patient never received antitumor therapy at the time of PD-L1 test. ^4^Retreatment: the relevant antitumor therapy for lung cancer, including chemotherapy, targeted therapy, immunotherapy, radiotherapy, and antitumor Chinese medicine therapy. ^5^Unknown: specific treatment options are not available to patients. ^6^Specimen storage duration: the duration from tissue sampling to the detection of PD-L1.

The article "Study on PD-L1 Expression in NSCLC Patients and Related Influencing Factors in the Real World" was retracted in 2023. Reasons: suspected computer-generated content; unreliable results or conclusions; concerns about the data; concerns about the results or conclusions.

**Table 4:** Correlation between pathological types of patients and tumor PD-L1 expression.

	PD‐L1 < 1% (*n* = 79)	1% ≤ PD‐L1 < 50% (*n* = 147)	PD‐L1 ≥ 50% (*n* = 70)	*P* value	OR
Pathologic types				0.014	Fisher
SCC	26 (33%)	83 (56%)	38 (54%)		
ADC	49 (59%)	58 (39%)	28 (39%)		
Others^∗^	5 (6%)	6 (4%)	5 (7%)		

SCC: squamous cell carcinoma; ADC: adenocarcinoma. ^∗^Other non-small-cell lung cancer except squamous cell carcinoma and adenocarcinoma.

**Table 5:** PD-L1 detection techniques for different immunotherapy agents.

Drug	Mechanism	Company	PD-L1 detection technology	Thresholds in clinical studies
Atezolizumab	PD-L1	Roche	Ventana PD-L1 (SP142) assay	TC0/1/2/3 or IC0/1/2/3
Avelumab	PD-L1	EMD	Without testing	1% or higher
Durvalumab	PD-L1	AstraZeneca	Ventana PD-L1 (SP263) assay	25% or higher
Pembrolizumab	PD-1	Merck	Dako PD-L1 IHC 22CS pharmDx	1% or 50% or higher
Nivolumab	PD-1	BMS	Dako PD-L1 IHC 28-8 pharmDx	≥1% or ≥5% or ≥10%

## Data Availability

The data used to support the findings of this study are included within the article.
